The article "Neutrophil–lymphocyte ratio (NLR) was associated with prognosis and immunomodulatory in patients with pancreatic ductal adenocarcinoma (PDAC)" was published in 2020. Journal: Biosci Rep.

# Neutrophil–lymphocyte ratio (NLR) was associated with prognosis and immunomodulatory in patients with pancreatic ductal adenocarcinoma (PDAC)

**DOI:** 10.1042/BSR20201190

**Published:** 2020-06-17

**Authors:** Zi-jun Xiang, Tao Hu, Yun Wang, Hao Wang, Lin Xu, Ning Cui

**Affiliations:** 1 Center of Liver-Biliary-Pancreatic, Taihe Hospital, Shiyan City, Hubei Province, China; 2 Department of Radiology, Zhuxi People's Hospital, Shiyan City, Hubei Province, China; 3 Medical Imaging Center-Intervention Room, Taihe Hospital, Shiyan City, Hubei Province, China

**Keywords:** Neutrophil-lymphocyte ratio, pancreatic cancer, prognosis

## Abstract

Although the oncological outcomes in patients with pancreatic ductal adenocarcinoma (PDAC) have markedly improved over the past decade, the survival prediction is still challenging. The aim of this study was to investigate the prognostic value of neutrophil–lymphocyte ratio (NLR) and analyze the relationship of between the NLR and immune cells phenotypes in patients with PDAC. Sixty-seven consecutive patients with PDAC were recruited in this study. Life-table estimates of survival time were calculated according to the Kaplan and Meier methodology. The phenotypic T cells subclasses were evaluated by flow cytometry. All the 67 patients in this study were treated with surgical resection and among them, 46 patients received adjuvant chemotherapy. Receiver operating characteristic (ROC) curves analysis was performed to compare prognostic value of NLR with CA199. We found that the Harrell's area under ROC (AUROC) for the NLR to predict overall survival (OS) (0.840; 95% CI, 0.766–0.898) was significantly higher than that of the CA199 levels. After that we stratified all patients into NLR > 2.5 (*n* = 42) and NLR ≤ 2.5 (*n* = 25) groups according to the OS of patients with PDAC. Survival analysis showed that patients with NLR ≤ 2.5 had significantly favorable OS and progressive free survival (PFS) compared with patients with NLR > 2.5. The CD3+ and CD8+/CD28+ T cell subsets were significantly increased in patients with NLR ≤ 2.5 (*P*<0.05), while the CD8+/CD28- and CD4+/CD25+ cell subsets were significantly decreased in patients with NLR ≤ 2.5 (*P*<0.05). In conclusion, a high NLR value independently predicts poor survival in patients with PDAC after surgical resection. The NLR was closely related with immune cells phenotypes The NLR may help oncologists evaluate outcomes of patients received surgical resection and chemotherapy to choose alternative therapies for patients with high NLR value.

## Introduction

Pancreatic ductal adenocarcinoma (PDAC), one of the most common cancers with high degree of malignancy, is a devastating disease all over the world [1–3]. Although the oncological outcomes in patients with PDAC have markedly improved over the past decade, the survival prediction is still challenging [4,5]. A large proportion of patients are diagnosed at advanced stage in the world, which would be the leading cause of cancer-related mortality. the median survivals for those patients with metastatic diseases were 6–12 months [6,7]. Surgical resection is the common and main treatment for patients with PDAC. Although mortality rates following pancreatectomy are now less than 5% in high-volume tertiary referral centers, morbidity following pancreatectomy is still common with rates estimated as high as 40–50% [8,9]. Currently, oncological outcomes in patients with advanced PDAC have markedly improved with multimodal neoadjuvant treatment (NAT) followed by surgical resection and NAT followed by surgery was regard as the guideline treatment for patients with PDAC [10–12].

The article "Neutrophil–lymphocyte ratio (NLR) was associated with prognosis and immunomodulatory in patients with pancreatic ductal adenocarcinoma (PDAC)" was published in 2020. Journal: Biosci Rep.

Carcinoembryonic antigen, carbohydrate antigen 15-3 (CA15-3), carbohydrate antigen 19-9 (CA19-9) and carbohydrate antigen 125 (CA125), and carcinoembryonic antigen (CEA) are routinely used in clinical practice to make diagnostic prevalence, determine prognosis and monitor therapeutic responses in gastroenterological cancers. Among these, the most common and best-identified marker for pancreatic cancer is CA19-9 [13]. Previous studies also showed that serum CA125 and CEA are important tumor biomarkers for the early diagnosis of pancreatic cancer [14,15].

Inflammatory response plays a vital role in tumor progression including initiation, promotion, malignant conversion, invasion, and metastasis [16,17]. Based on these factors, several inflammations and immune-based prognostic scores such as lymphocyte count, platelet–lymphocyte ratio (PLR), and neutrophil–lymphocyte ratio (NLR) have been developed to predict the inflammatory response being associated with poor survival and recurrence in different types of cancer, including PDAC [18–20]. An increasing body of evidence shows that systemic inflammation activation exerted by cancer cells anticipates tumor progression *via* inducing cancer proliferation and metastasis or promoting angiogenesis [21,22].

However, the previous studies have deficiencies that these indexes did not comprehensively reflect the balance of host inflammatory and immune status. Challenges remain in order to identify reliable, cost-effective biomarkers to identify which patients are most likely to receive therapeutic benefit from pancreatectomy. In the present study, we evaluated the prognostic value of NLR in patients with pancreatic cancers who received surgical resection. Moreover, we also analyzed the relationship of between the NLR and immune cells phenotypes and other clinical characteristics.

The article "Neutrophil–lymphocyte ratio (NLR) was associated with prognosis and immunomodulatory in patients with pancreatic ductal adenocarcinoma (PDAC)" was published in 2020. Journal: Biosci Rep.

## Patients and methods

### Study design and participants

The cohort consisted of 67 consecutive patients with PDAC identified retrospectively from January 1, 2014 to August 30, 2018. The study was approved by the Regional Ethical Review Board for Center of Liver-Biliary-Pancreatic, Taihe Hospital, Shiyan City. The IRB number of this study is TH032915. Patients were treated according to the Declaration of Helsinki's ethical principles for medical research involving human subjects. All patients provided an informed written consent prior to study entry. Patients were required to meet the following inclusion criteria: participants were age 18–80 years; Eastern Cooperative Oncology Group performance status (ECOG-PS) [23] was evaluated; the primary procedure was surgical resection, histologically or cytologically confirmed PDAC. No prior chemotherapy or immunotherapy was allowed. Patients were excluded if they had a concurrent malignancy other than PDAC, a serious, uncontrollable medical condition, or a psychiatric disorder that would limit ability to comply with study requirements.

### Pretreatment evaluation

Medical history and physical findings were documented in each patient. Each patient also had an electrocardiogram (ECG), computed tomography of the abdomen and pelvis (and thorax, if needed), serum chemistry and complete blood count (CBC), and urine analysis.

### Procedures

All patients received surgical resection, while 46 patients received adjuvant chemotherapy and number of previous lines of palliative intent chemotherapy were recorded. Adverse events were assessed according to the National Cancer Institute's Common Terminology Criteria for Adverse Events version 4.0 (NCI-CTCAE v4.0) and response to treatment was assessed by the Response Evaluation Criteria in Solid Tumors (www.cancer.gov/).

### Analysis of the circulating immune response

Peripheral venous blood was obtained from each patient before surgery. Most of the patients were collected at the second day of admission. Whole blood (100 ml) was incubated in the dark with primary antibody at 4°C for 15 min. Anti-CD3-FITC/anti-CD56-RPE (Dako), anti-CD3-FITC (fluorescein isothiocyanate), anti-CD4-RPE, anti-CD8-RPE, anti-CD45RO and anti-CD4-FITC/anti-CD25-PE (BD Biosciences) were used. After hemolysis for 10 min, samples were centrifuged for 10 min at 1500 rpm at room temperature, and then washed twice in PBS and subjected to flow cytometric analysis. Three-color flow cytometric analysis was performed to determine cell phenotypes using an FC500 (Beckman–Coulter) and CXP analysis software (Beckman–Coulter). Lymphocytes were gated by forward scatter versus side scatter. Analysis was set to collect 5000 gated events.

The article "Neutrophil–lymphocyte ratio (NLR) was associated with prognosis and immunomodulatory in patients with pancreatic ductal adenocarcinoma (PDAC)" was published in 2020. Journal: Biosci Rep.

### Statistical methods

Continuous variables were expressed as mean ± SD (standard deviation) and compared using a two-tailed unpaired Student's *t* test; categorical variables were compared using χ^2^ or Fisher analysis. The predictive performance of NLR was measured using the area under receiver operating characteristic (AUROC) [24]. Life-table estimates of survival time were calculated according to the Kaplan and Meier methodology [25]. The Greenwood formula was used for the standard deviation. A Cox proportional hazards regression approach [26] was chosen for the evaluation of overall survival (OS) and progressive free survival (PFS) as the primary end-point. Potential prognostic variables were analyzed both univariately with one factor taken at a time, and then in a multivariate model combining all factors. Results are reported as hazard ratios (HR) and their 95% confidence intervals (CI). An HR > 1 indicated an elevated risk with respect to the reference category. A confidence interval which did not include the value 1 indicated statistical significance at the 5% level. All statistical evaluations were carried out using SPSS software (Statistical Package for the Social Science, version 15.0, SPSS Inc, Chicago, IL). A value of *P*<0.05 was considered to be statistically significant in all the analyses.

## Results

### Patients’ characteristics

The 67 patients in this study were treated with surgical resection and 46 patients received adjuvant chemotherapy. Among these patients, 30 patients received FOLFIRINOX and 16 patients received nab-paclitaxel combined with gemcitabine. Patients received blood routine tests at multiple time points. Characteristics of all patients are detailed in Table 1.

**Table 1:** Demographics and clinical characteristics of all patients

Variable	NLR > 2.5 (*N* = 42)	NLR ≤ 2.5 (*N* = 25)	*P* values
**Age**	62.3 ± 11	65.4 ± 10.4	0.244
**Gender**			
**Female**	20	10	0.825
**Male**	22	15	
**ECOG-PS**			0.529
**1**	37	22	
**2**	5	3	
**TNM staging**			0.267
**I–II**	36	5	
**III**	6	24	
**Adjuvant chemotherapy**			0.178
**FOLFIRINOX**	20	10	0.373
**Nab-paclitaxel combined with gemcitabine**	10	6	
**Estimated blood loss (ml)**	1198.6 ± 863.3	1253.4 ± 943.3	0.352
**Tumor size (cm)**	2.58 ± 3.24	2.49 ± 4.56	0.426
**Neural invasion**			
**Yes**	24	15	0.763
**No**	18	10	
**Vascular invasion**			0.529
**Yes**	12	7	
**No**	30	18	
**CA-199**			0.684
**>12000**	29	18	
**<12000**	13	7	

### Comparison of prognostic value of NLR with CA199

We then performed ROC curves analysis to comparison prognostic value of NLR with CA199. We found that the Harrell's AUROC for the NLR to predict OS (0.840; 95% CI, 0.766–0.898) was significantly higher than that of the CA199 levels (0.694; 95% CI, 0.609–0.771; *P* = 0.001, Figure 1A). The NLR to predict PFS (0.720; 95% CI, 0.636–0.794) was significantly higher than that of the CA199 levels (0.598; 95% CI, 0.509–0.682; *P* = 0.007, Figure 1B). After that we stratified all patients into NLR > 2.5 (*n* = 42) and NLR ≤ 2.5 (*n* = 25) groups according to the prognosis of patients with PDAC.

The article "Neutrophil–lymphocyte ratio (NLR) was associated with prognosis and immunomodulatory in patients with pancreatic ductal adenocarcinoma (PDAC)" was published in 2020. Journal: Biosci Rep.

**Figure 1:** Survival prediction comparison (**A**) AUROC of NLR and CA199 in predicting OS; (**B**) AUROC of NLR and CA199 in predicting PFS.

### Survival analysis of patients with PDAC with respect to NLR

In present study, we found that OS (*P* = 0.018, Figure 2A) and PFS (P = 0.033, Figure 2B) in the NLR ≤ 2.5 group were significantly better than those in the NLR > 2.5 group. The stratified analysis found that patients with NLR ≤ 2.5 in the chemotherapy treatment group had significantly different OS (*P* = 0.032, Figure 3A) and PFS (*P* = 0.031, Figure 3B) than patients with NLR > 2.5, and had significant survival advantages. In the group without chemotherapy, there was no significant difference in OS (*P* = 0.213, Figure 3C) and PFS (*P* = 0.562, Figure 3D) between patients with NLR ≤ 2.5 and patients with NLR > 2.5.

**Figure 2:** Survival analysis (**A**) OS and (**B**) PFS for the different groups divided by NLR.

**Figure 3:** Survival stratification (**A**) Overall survival and (**B**) progression free survival for patients with chemotherapy. (**C**) Overall survival and (**D**) progression free survival for patients without chemotherapy.

### Predictors associated with clinical outcomes

Cox proportional hazards models were then used to quantify the prognostic significance of risk factors after multivariable adjustment. A multivariable analysis was performed to assess the factors that demonstrated significant effects in univariate analysis. After adjusting for competing risk factors, NLR ≤ 2.5 (HR: 2.104, 95% CI: 1.582–4.372, *P* = 0.003), vascular invasion (HR: 1.318, 95% CI: 1.221–3.149, *P* = 0.032) and CA199 levels (HR: 1.303, 95% CI: 1.147–2.659, *P* = 0.012) remained independent predictors of PFS and OS. The details are shown in Table 2.

**Table 2:** Multivariable Cox proportional hazard regression analysis of patients' clinical characteristics and survival

Variables	PFS		OS	
	HR (95% CI)	*P* value	HR (95% CI)	*P* value
ECOG-PS: 2	1.087 (0.716–1.358)	0.562	0.873 (0.761–1.132)	0.833
TNM staging:III	1.003 (0.882–1.132)	0.638	0.944 (0.839–1.241)	0.793
NLR ≤ 2.5	1.725 (1.448–3.103)	0.027	2.104 (1.582–4.372)	0.003
Vascular invasion	1.424 (1.199–1.219)	0.004	1.318 (1.221–3.149)	0.032
CA199 levels	1.383 (1.127–2.639)	0.001	1.303 (1.147–2.659)	0.012

The article "Neutrophil–lymphocyte ratio (NLR) was associated with prognosis and immunomodulatory in patients with pancreatic ductal adenocarcinoma (PDAC)" was published in 2020. Journal: Biosci Rep.

### Phenotypic analysis of peripheral blood immune cells

Phenotypic analysis of peripheral blood mononuclear cells: CD3 + and CD8 + / CD28 + T cell subsets were significantly increased in patients with NLR ≤ 2.5 before treatment and after the end of the first cycle (*P*<0.05), CD8 + / CD28- and CD4 + / CD25 + cell subsets were significantly reduced (*P*<0.05) (Figure 4A–F). In the NLR > 2.5 group, only the CD3 + T cell subsets were significantly increased (*P*<0.05).

**Figure 4:** Peripheral blood T cell phenotype measurements via cytometry before and after the operations (**A–F**) Subtypes of T cell phenotype from patient's peripheral blood.

## Discussion

Despite of the improvement in the treatment outcomes of most malignant tumors, the treatment outcome for pancreatic cancer remains dismal. One of the reasons for extremely poor survival outcome in pancreatic cancer is that only 15–20% of patients are diagnosed early enough for it to be resectable [27,28]. Researchers reported the results of a highly effective fluorouracil plus leucovorin, irinotecan, oxaliplatin (FOLFIRINOX) treatment in patients with metastatic pancreatic cancer that led to a major change in the therapeutic paradigm in patients with advanced pancreatic cancer [29,30]. In addition to chemotherapy, there are several treatment modalities including radiotherapy, immunotherapy, adoptive cell therapy and cancer vaccines. Recently, a clinical study used treatment of combined adoptive cells infusions and chemotherapy and proved that it was safe, and resulted in favorable PFS and OS [31].

The NLR, which has been considered as a member of the marker of the systemic inflammation response, is valuable for predicting the prognosis of various cancers [32–34]. This study showed that assessment of the NLR calculated from CBCs before treatments predicted prognosis of patients with PDAC independently. The result is consistent with previously published papers displaying that high NLR with poor outcome in patients with pancreatic cancers [35,36]. Yet, the cutoff values of the NLR were inconsistent in these above studies, which reduces its clinical applicability. We rethought the impact of the NLR and explored it as a continuous explanatory variable that affected by the patients baselines and therapeutic approaches. Consequently, we found that the pretreatment value of 2.5 was the most appropriate cutoff value and not only the statistical sensitivity and specificity were taken into account but also the clinical significance. Our data indicated that the median OS of patients in NLR > 2.5 group was much shorter when compared with those in NLR ≤ 2.5 group.

The article "Neutrophil–lymphocyte ratio (NLR) was associated with prognosis and immunomodulatory in patients with pancreatic ductal adenocarcinoma (PDAC)" was published in 2020. Journal: Biosci Rep.

The mechanism underlying the potential prognostic value of NLR is mainly due to the significance of the infiltrated neutrophils and lymphocytes. The systemic inflammatory response from cancer cells promotes the infiltration of neutrophils, which benefits cancer progression via secreting interleukin-2 (IL-2), interleukin-6 (IL-6), interleukin-10 (IL-10), tumor necrosis factor α (TNF-α) and vascular endothelia growth factor (VEGF) [37,38]. VEGF is a proangiogenic factor contributes to cancer development especially through angiogenesis. Moreover, increased TNF-α and IL-10 issue in lymphocyte count decrease and lymphocyte dysfunction also [39].

By the way, there were several limitations of this study: on one hand, this is a study with small sample size and retrospective design. On the other hand, the relationship between survival and change of NLR after treatment apart from pretreatment can be investigated in future studies.

In conclusion, a high NLR value independently predicts poor survival in patients with PDAC after surgery. The NLR may help oncologists evaluate outcomes of patients received surgical resection and chemotherapy in order to choose alternative therapies for patients with high NLR value.

## Abbreviations

AUROC: area under ROC
CBC: complete blood count
IL-2: interleukin-2
NAT: neoadjuvant treatment
NLR: neutrophil–lymphocyte ratio
OS: overall survival
PDAC: pancreatic ductal adenocarcinoma
PLR: platelet–lymphocyte ratio
PFS: progressive free survival
ROC: receiver operating characteristic
TNF-α: tumor necrosis factor α
VEGF: vascular endothelia growth factor
